The article "A Convolutional Neural Network-Based Model for Supply Chain Financial Risk Early Warning" was retracted in 2023. Reasons: signs of a paper mill; suspected computer-generated content; unreliable results or conclusions; concerns about the data.

# A Convolutional Neural Network-Based Model for Supply Chain Financial Risk Early Warning

**DOI:** 10.1155/2022/7825597

**Published:** 2022-04-15

**Authors:** Li-Li Yin, Yi-Wen Qin, Yuan Hou, Zhao-Jun Ren

**Affiliations:** ^1^Beijing Technology and Business University, Beijing, China; ^2^North Borneo University College, Kota Kinabalu, Sabah, Malaysia

## Abstract

At present, there are widespread financing difficulties in China's trade circulation industry. Supply chain finance can provide financing for small- and medium-sized enterprises in China's trade circulation industry, but it will produce financing risks such as credit risks. It is necessary to analyze the causes of the risks in the supply chain finance of the trade circulation industry and measure these risks by establishing a credit risk assessment system. In this article, a supply chain financial risk early warning index system is established, including 4 first-level indicators and 29 third-level indicators. Then, on the basis of the supply chain financial risk early warning index system, combined with the method of convolution neural network, the supply chain financial risk early warning model of trade circulation industry is constructed, and the evaluation index is measured by the method of principal component analysis. Finally, the relevant data of trade circulation enterprises are selected to make an empirical analysis of the model. The conclusion shows that the supply chain financial risk early warning model and risk control measures established in this article have certain reference value for the commercial circulation industry to carry out supply chain finance. It also provides guidance for trade circulation enterprises to deal with supply chain financial risks effectively.

## 1. Introduction

The commercial circulation industry is a comprehensive industry composed of enterprises specializing in the circulation of all kinds of commodity trade and providing services for the circulation of commodity trade, mainly including commodity wholesale and retail, storage, transportation, and other sectors [1, 2]. Commercial circulation enterprises play a connecting role in the process of the development of China's market economy, and the goods produced by production enterprises reach the hands of consumers through logistics distribution. The commercial circulation industry is one of the most important basic links in the production and economic activities of the market economy society [3]. In recent years, even under the background of the “new normal,” China's commercial circulation industry has maintained good development momentum, with the industry output increasing year by year. However, the commercial circulation industry also faces bottlenecks hindering its development and progress. The reason is the existence of difficult financing and expensive financing problems. The commercial circulation industry must further develop to solve these problems, which has become a top priority.

In the traditional financing mode, commercial circulation enterprises cannot effectively solve the structural problems of financing difficulties for small- and medium-sized enterprises, and it is difficult to obtain a large amount of funds for enterprise operation and development [4, 5]. At present, there are several substantial problems in China's traditional financing mode. The first problem in the development of commerce is that there is an important indirect financing mode, namely, the money supply main body for the financing model of commercial banks. However, the financing pattern also has disadvantages, such as the high-level requirements for financing companies, relatively high financing prices, and low financing efficiency, making most small and medium circulation enterprises unable to obtain funds from commercial banks. In addition, the financing difficulties of commercial circulation enterprises are related to other factors, including the development trend of China's commercial circulation industry and risk preference management within commercial banks [6, 7]. Second, as China has not yet perfected its capital market regulatory system, financing risks exist, leading to the inability of most small- and medium-sized enterprises in commercial circulation to adopt a direct financing mode [8, 9]. Third, there is also a kind of financing model of financing efficiency that is high, namely, small loan companies, P2P platforms, and private lending and financing, but because of considerable potential safety problems, financing in this manner is also more expensive. This approach has had a bad effect on China's existing financial markets and has been unable to solve the financing problem [10, 11].

Two reasons for these problems are summarized through analysis. First, in the current financial environment in China, the financing risk control mechanism of traditional banks and other financial institutions for small- and medium-sized financing enterprises is sufficient. From the perspective of commercial banks, commercial banks must strengthen risk control measures to ensure that enterprises have a strong ability to handle default risks when risk problems occur in the process of financing and to recover losses. Moreover, the information provided by financing enterprises to commercial banks and other financial institutions may not be entirely accurate. Even without the existence of moral hazard, commercial banks will strengthen risk control measures. Commodity trade financing is an important part of commercial circulation enterprises. However, due to the existence of information asymmetry, commercial banks sometimes fail to ensure the authenticity of transactions of financing enterprises, thereby raising doubt among financing enterprises and reducing financing efficiency. Second, in the context of the “new normal” of the economy, enterprises are faced with a severe environment, such as macroeconomic changes and unbalanced industrial structure, which makes it difficult to survive and develop. From the perspective of commercial circulation enterprises, small and medium enterprise (SMEs) in the supply chain do not have enough financial support due to limited operation and development. In the supply chain do not have sufficient financial support due to limited operation and development. If enterprises have problems in the operation process, it will affect the repayment of bank debts. Therefore, such enterprises cannot easily obtain financing from commercial banks. However, most commercial circulation enterprises are small in scale and uneven in level, with many unstable factors that are easily affected by the operating environment and operating conditions. Therefore, financing is difficult to obtain via the traditional financing mode. If these SMEs in the supply chain are considered, they can guarantee that core enterprises resolve risks from the perspective of the supply chain, rather than being shut out by commercial banks due to problems such as insufficient solvency and high market risk. Therefore, it is very necessary to establish a risk warning mechanism in the online supply chain finance carried out in the commercial circulation industry, which can play a role before the risk occurs and achieve the purpose of risk prevention. As the trade circulation industry is an industry with small- and medium-sized enterprises as the main body, the number of these enterprises is huge, but the management level is relatively low. In the supply chain, the relationship between enterprises is close, and the possibility of problems in the operation process of these small- and medium-sized enterprises is relatively large. Under the joint action of these factors, once a risk occurs, it will affect all participating enterprises. In addition, the online supply chain finance of the commercial circulation industry is jointly promoted by the B2C e-commerce platform and commercial banks, and the cooperation between all participating enterprises. In the supply chain, each enterprise is not a simple and independent individual, and various problems in the operation process will directly or indirectly affect the operation and development of other enterprises, in turn affecting the whole supply chain. Therefore, each enterprise should coordinate with each other and adjust each other. In the early warning of risks, while controlling their own risks, they must consider the interests of other participating enterprises. Coordinated alarm is an effective measure to control and prevent risks. It is necessary to analyze the causes of supply chain finance risks in commercial circulation industry and measure these risks by establishing credit risk assessment system.

## 2. Literature Review

### 2.1. The Development of Supply Chain Finance

China's supply chain finance originated from the “1+N” mode proposed by Shenzhen Development Bank. Later, domestic commercial banks began to provide supply chain finance services. After years of development, this mode has become an important way for enterprises to obtain financing [12–14]. Supply chain finance can fundamentally solve the financing dilemma of commercial circulation enterprises, control risks from the whole supply chain, reduce other risks, and provide a good direction for the transformation and development of the commercial circulation industry [15]. Over time, in the context of Internet finance, China's commercial circulation enterprises have formed many supply chain finance business models through continuous development and innovation, such as the supply chain financing model with Alibaba, JINGdong, and other e-commerce platforms as the core [16]. In China, supply chain finance can be divided into two categories: traditional supply chain finance [17] and new supply chain finance [18]. Traditional supply chain finance is dominated by commercial banks and other financial institutions. By providing supply chain financial services, banks can closely link core enterprises and their upstream and downstream enterprises with third-party logistics enterprises and other supply chain participants, and meanwhile reduce financial risks of banks [19].

With the rapid development of the Internet and the integration of technology, the business model of supply chain finance begins to go online and the information sharing degree is higher [20]. It can not only solve the problems existing in the traditional financing mode but also enhance the connection between various enterprises in the supply chain. After continuous development and innovation, Internet financial platforms have formed different types of supply chain finance business models [21], which can be summarized as supply chain finance model based on B2B e-commerce platform, supply chain finance model based on B2C e-commerce platform, supply chain finance model based on payment, and other models. Later, the addition of big data and cloud computing technology changed the traditional supply chain finance model, which can collect information more accurately, thus reducing the occurrence of credit risk. also facilitates transactions between enterprises, increases development opportunities, and reduces transaction costs, creating a good financial environment for the development of enterprises in the whole supply chain.

### 2.2. Risk Identification of Supply Chain Finance

Scholars domestically and abroad have extensively studied how to conduct supply chain finance and use these business models to effectively identify risks. Mou et al. [22] stated that commercial banks should combine immovable property mortgage and chattel ownership pledge loans to ensure the normal circulation of goods and capital when conducting supply chain finance business and that risks must be dispersed. Antonella et al. [23] found that supply chain finance models play an important role in the development of commercial banks. They analysed various models, identified and assessed credit risks and presented suggestions for the credit risk management of supply chain finance. Abbasi et al. [24] studied the accounts receivable financing mode and probed credit risk evaluation. They found that previous supply chain financial risk management has been unable to avoid risk. However, from the perspective of the supply chain, they analysed the relationship between each participating main body and concluded that there exists a relationship of cooperation. The ability of enterprises to avoid risks can be consolidated, which is beneficial to the development of supply chain finance. Szopinski [25] conducted an in-depth analysis of the main reasons for the credit risks of SMEs in the e-finance of the online commercial financing bank online supply chain, established a credit risk analysis framework, and invited experts to suggest effective prevention methods to address the credit risks of SMEs in the e-finance of the online commercial financing bank online supply chain. Lahkani et al. [26] believed that for Internet third-party B2B e-commerce, if the credit and financial status of SMEs are not improved, continuous deterioration and increases in the credit risks of SMEs may occur. Based on the third-party B2B e-commerce platform, Thatcher et al. [27] established an index system for the credit risk evaluation of commercial financing banks in the online third-party supply chain provided by SMEs and applied a multilevel grey credit evaluation model to comprehensively evaluate the actual credit and financial status of SMEs with third-party loans. The application feasibility of the grey evaluation model is verified via an example. Montes et al. [28] reported an analysis of online supply chain finance security and credit risk and proposed strategies to address credit risk.

### 2.3. The Model Application of Supply Chain Financial Risk Warning

Scholars domestically and abroad have begun to use the new nonlinear research model analysis method to analyze small- and medium-sized enterprise supply chain marketization financial risk [29]. Yang et al. [30] established a supply chain financial risk management model under the Internet finance mode. An Internet supply chain financial risk management model based on data science was proposed to improve the supply chain's ability to resist risk. On the basis of studying supply chain finance and risk-related theories, Fan [16]used fuzzy preference relations to select the main risk criteria and constructed a risk evaluation index system. From the perspective of optimizing the supply chain finance mode, Sun [31] designed a new inventory pledge financing mode that combines the functions of Internet of things technology and the characteristics of the supply chain finance inventory pledge financing mode. Bandaly et al. [32] established a stochastic optimization model for supply chain operation and financial risk management. Based on this model, the performance of the integrated risk management model (in which operational risk management decisions and financial risk management decisions are made simultaneously) and the sequential model (in which financial risk management decisions are made after the operational risk management decisions are finalized) are compared.

In view of the above problems in the research, to further study supply chain finance risk and financial risk early warning modelling framework and to build a supply chain through the establishment of a relatively complete risk identification risk evaluation index system, this article uses principal component analysis and a convolution neural network model. Additionally, empirical analysis is used to verify the validity of the model. Thus, this novel approach can provide theoretical support for the early warning of supply chain finance risk and the development of supply chain finance business in the commercial circulation industry.

## 3. Research Design

### 3.1. Design Ideas for the Index System

In the supply chain financial risk early-warning evaluation index system established by existing scholars, indicators related to the qualification of finance enterprises [33, 34], such as profitability and debt paying ability, have been thoroughly studied, so little room for innovation remains. However, from the perspective of the whole supply chain, analysis of the indicators of risk is relatively understudied, not only to the development status of the financing enterprise but also to the management research. More financing enterprises and factors in the supply chain must be considered, including changes in the macro environment, the qualification status of the core enterprise, and the pledges and relationships among all the main participants in supply chain finance. In this way, the factors affecting supply chain finance risk can be comprehensively analysed, and an effective evaluation index system can be established to reflect the overall risk characteristics of supply chain finance.

The design idea of the index system is shown in Figure 1.

Therefore, this article first analyses the financing mode of the supply chain finance of the commercial circulation industry and identifies the factors influencing risk. On the basis of the existing credit risk assessment index system and using the “main body + debt” credit analysis structure, we design a comprehensive supply chain financial risk early warning index system. The credit rating of small- and medium-sized enterprises in the commercial circulation industry should be assessed accurately, and the degree of risk should be given as an early warning. Moreover, supply chain finance should be better developed to reduce the financing difficulties faced by these enterprises.

### 3.2. Basic Structure of the Index System

The influencing factors of risk are identified through the above process analysis of the supply chain finance mode of the commercial circulation industry. Then, referring to the related literature on the construction of risk early warning index systems [35, 36], we eliminated some difficult quantitative indicators. Finally, the core enterprise financing business qualifications, environmental conditions, the characteristics of the qualification, and the supply chain operating conditions are used to establish a risk early-warning index system that contains three levels and 29 indicators.

The risk early-warning indicator system and its description are shown in Table 1:

## 4. Research Method

### 4.1. Principal Component Analysis

Principal component analysis is a multivariate statistical analysis method. Through the linear combination of multiple original variables, several principal component variables that can reflect most of the information of the original variables are derived [37].

The main calculation steps of principal component analysis are as follows:

The first step is to standardize the original index data.

First, the selected index data are constructed into a matrix *X*, as shown in formula (1).

(1) $$\begin{array}{c} X=\begin{array}{cccc} x_{11} & x_{12} & \cdots & x_{1p}\\ x_{21} & x_{22} & \cdots & x_{2p}\\ \vdots & \vdots & \vdots & \vdots \\ x_{n1} & x_{n2} & \cdots & x_{\text{np}} \end{array}. \end{array}$$

Then, a standardized matrix *Z* is obtained by standardizing matrix *X*. The process eliminates the impact of data due to the disunity of index quantification methods, as shown in formula (2).

(2) $$\begin{array}{c} Z_{\text{ij}}=\frac{x_{\text{ij}}-{\bar{x}}_{j}}{\sqrt{\text{var}\left(x_{j}\right)}}\;\left(i=1,2,\ldots ,n;j=1,2,\ldots ,p\right). \end{array}$$

In formula (2), ${\bar{x}}_{j}=1/n\sum_{1}^{n}x_{\text{ij}}$, $\text{var}\left(x_{j}\right)=1/n-1\sum_{1}^{n}{\left(x_{\text{ij}}-{\bar{x}}_{j}\right)}^{2},\left(j=1,2,\ldots ,p\right).$

The second step is to solve the correlation coefficient matrix of the matrix *Z* obtained in the previous step, as shown in formula (3).

(3) $$\begin{array}{c} R=\left[r_{\text{ij}}\right]\text{xp}=\frac{Z^{T}Z}{n-1}. \end{array}$$

In the formula, *r*_ij_=1/*n* − 1∑_*t*−1_^*n*^*x*_ti_*x*_tj_(*i*, *j*=1,2,…, *p*).

The third step is to solve the correlation coefficient matrix *R* and obtain the eigenvalues and the eigenvectors corresponding to each eigenvalue. According to the knowledge of linear algebra, *p* characteristic roots can be solved by using the formula *R* − *λI*_*p*_=0, and then the eigenvalue (*λ*_1_, *λ*_2_,…, *λ*_*p*_) of the correlation coefficient matrix and the corresponding eigenvector *a*_*i*_=(*a*_*i*1_, *a*_*i*2_,…, *a*_ip_) of each eigenvalue can be calculated.

The fourth step is to use the standardized index variables to write the expressions of the principal component variables, as shown in formula (4).

(4) $$\begin{array}{c} F_{p}=a_{1i}Zx_{1}+a_{2i}Zx_{2}+\cdots +a_{\text{pi}}{\text{Zx}}_{p}. \end{array}$$

In the formula, *F*_*p*_ represents the Pth principal component, *a*_1*i*_, *a*_2*i*_,…, *a*_pi_ denote the eigenvectors corresponding to the eigenvalue of the covariance matrix of *X*, and *Zx*_1_, *Zx*_2_,…, Zx_*p*_ represents the standardized value of the original variable.

Finally, the extracted principal components are evaluated comprehensively. Taking the contribution rate of variance as the weight, the final evaluation value can be obtained by weighted summation of *k* principal component variables.

### 4.2. Convolutional Neural Network

The convolutional neural network model (CNN) is a representative deep learning algorithm [38]. It is actually a feedforward neural network with a deep structure. In contrast to traditional neural networks, CNNs have neural network structures that are not completely connected.

The hidden layer of the convolutional neural network can be divided into three parts: a convolutional layer, a pooling layer and a fully connected layer. One part performs feature extraction, and the other part is responsible for classification recognition. By means of a convolution kernel and translation, each layer of neurons is connected locally to achieve hierarchical feature extraction and transformation of input data. Neurons with the same connection weight are connected to different areas of the neural network of the previous layer, and a neural network structure with unchanged properties is obtained, as shown in Figure 2.

#### 4.2.1. Convolution Process

The input data of the model are first imported into the convolution layer, and the function of the convolution layer is to extract features from these data. The convolution kernel is an important concept in the calculation of the convolution layer. It is composed of many elements, and each element has its corresponding weight coefficient and corresponding deviation. Multiple such convolution kernels constitute the input object. Another concept is the neuron; a convolution layer has many neurons. Each neuron is connected to multiple neurons in the previous layer. The specific number of neurons is closely related to the size of the convolution kernel and plays a decisive role. The main feature that can be extracted from the convolution layer is the function of the convolution kernel. Specifically, the convolution kernel periodically scans the input features and multiplies the input features in the perception domain and matrix elements to obtain the output features. The convolution kernel is the core of the convolution layer function, and the original features are calculated by means of the inner convolution operation of the matrix and the summation operation of the offset layer, as shown in formula (5). If different convolution kernels are used for repeated calculation, a series of different output features can be obtained.

(5) $$\begin{array}{c} X_{j}^{\int^{}}=f\left(\sum_{i\in p_{j}}X_{i}^{\int^{}-1}K_{\text{ij}}^{\int^{}}+b_{j}^{\int^{}}\right). \end{array}$$

In the calculation process, in general, the eigenmatrix or vector selected on the feature can be used to determine the corresponding position of the i-th convolution kernel on the input feature, represented by *p*_*j*_ in the formula. *X*_*i*_^∫−1^ represents the corresponding value of the input feature at the first layer, and *X*_*j*_^∫^ is the corresponding value of the output feature at the first layer obtained after the convolution operation. *K*_ij_^∫^ is the corresponding weight value of each element in the convolution kernel. *b*_*j*_^∫^ is the offset value of the feature, and each convolution layer and each pooling layer correspond to a offset value.

#### 4.2.2. Pooling Process

In the first step of the convolution process, new output features are extracted from the original features through calculation of the convolution kernel. The second step is to import these output characteristics into the pooling layer. In the pooling layer, these output features can be sampled; that is, feature selection and information filtering can be conducted on the output data of the convolution layer. Similar to the input data in the convolution layer, the input data in the pooling layer select the pooling region in the same way. This area is determined by the pooling size, step size, and population. The calculation process of the pooling layer is similar to that of the convolution process. The window size is set; then, the maximum or average value in the window area is selected as the characteristic value of the sliding window. In contrast to the output results obtained in the convolution layer, the pooled layer outputs the features after dimensionality reduction after the calculation. The specific process is shown in formula (6).

(6) $$\begin{array}{c} X_{j}^{\int^{}}=f\left(\text{pool}\left(X_{i}^{\int^{}-1}\right)+b_{j}^{\int^{}}\right), \end{array}$$

where *X*_*i*_^∫−1^ in the formula represents the input characteristics of layer ∫ − 1. *X*_*j*_^∫^ represents the corresponding value on the output characteristics of the ∫ layer. *K*_ij_^∫^ is the weight of the convolution kernel, and *b*_*j*_^∫^ represents the bias in features. Pool (^*∗*^) represents a maximum or average value function. The pooling process corresponds to the extraction process of features.

#### 4.2.3. Fully Connected Layer

Finally, there is a connection layer that connects the pooling layer to the multilayer perceptron, which has the same function as the hidden layer in traditional neural networks. In the CNN model, the connection layer is generally connected to the last part of the hidden layer of the network, which has a conduction effect and can transmit signals to other connection layers. In the connection layer, the output feature graph is converted into a vector or matrix and passed to the multilayer perceptron via an activation function.

In practical analysis, the initial input data pass through multiple convolution and pooling layers and extract features from the convolution layer as the input data into the pooling layer. This process is repeated to eventually obtain the results after several feature extractions. The formula of the fully connected layer is shown in formula (7).

(7) $$\begin{array}{c} X_{j}^{\int^{}}=f\left(U^{\int^{}}\right),\\ U^{\int^{}}=K^{\int^{}}X^{\int^{}-1}+b^{\int^{}}, \end{array}$$

where *f* (^*∗*^) is the activation function. *X*^∫−1^ is the layer ∫ − 1 input characteristic. *X*_*j*_^∫^ is the corresponding value on the output characteristics of ∫ layer. *K*^∫^ means to calculate the weight of layer ∫ − 1 to layer ∫. The final prediction results are obtained by connecting the features to the outputs through a complete connection layer.

#### 4.2.4. ReLU Activation Function

The rectified linear unit (ReLU) function is one a common activation functions, and its expression is shown in formula (8).

(8) $$\begin{array}{c} f\left(x\right)=\max\left(0,x\right). \end{array}$$

The ReLU function can sparsely activate neurons to better mine relevant features and fit training data. A CNN is a highly nonlinear model. For nonlinear functions, the gradient of the nonnegative interval of ReLU is constant, so there is no issue with vanishing gradients, and the convergence rate of the model is maintained in a stable state.

CNNs overcome the limitations of traditional linear prediction methods, can more accurately process qualitative and quantitative data in risk prediction indicators, and are less constrained by data quality. Moreover, CNNs can collect the essential characteristics of data sets from fewer samples, greatly reducing the number of training parameters in the network and the amount of calculation.

### 4.3. Model Initialization and Learning Rate Setting

First, the CNN model should be initialized such that each neuron is initialized into an effective state. For example, the tansig function has good nonlinearity in the range of [−1.7, 1.7], and the random initialization method can also set the initial values of parameters between [−1, 1]. By means of initialization, the input of the function and the initialization of the neuron can be within a reasonable range such that each neuron is valid at the time of initialization.

If the order of magnitude of the data is large, the gradient may be too large, and the solution speed of the model will be slow. Therefore, in the training process of the model, gradient descent is used to optimize the learning of parameters and accelerate the model to obtain the optimal solution. When the gradient descent method is used for training, the model is initialized first, and an initial value range is set for each parameter. As the selected index data are normalized in this article, the problem of neuron saturation caused by excessive order of magnitude will be avoided. Therefore, a random initialization method can be selected to set the initial parameters of the model, which is convenient for subsequent training.

Through the analysis of the relationship between the gradient and learning rate, it can be concluded that if the order of magnitude of each gradient is not the same, then the order of magnitude of the learning rate they need is not the same. The learning rate of model training should be set in an appropriate range to improve the performance of gDA. If the learning rate is too high, the gradient could disappear, making the training situation of the model unstable. If the learning rate is too small, gradient explosion may occur, resulting in a large decrease in the solving speed of the model. After data normalization, there is no need to adjust the learning rate according to the range of data. Therefore, an adaptive learning rate can effectively solve this problem. During the training process, the learning rate can be adjusted by simulated annealing, for example, by setting the initial learning rate to 0.1 and then multiplying the rate by a step factor of 0.9 in each subsequent training cycle. In this way, the model can not only improve the speed of obtaining the optimal solution but also achieve the desired training effect.

## 5. Results and Analysis

### 5.1. Data Sources and Processing

In this article, 80 commercial circulation enterprises are selected as samples, and the corresponding data of the financial indicators are derived from the database of Guotai 'an. “Whether an enterprise is an ST” is used as the evaluation standard of enterprise default. If an enterprise is an ST, the enterprise has a certain degree of risk of solvency, the debt repayment pressure is larger, and the risk is larger, which is not conducive to the long-term operation and development of the enterprise. Therefore, this value can be used to distinguish whether the enterprise defaults. In the sample data, 12 enterprises are identified as ST and are judged to be in default, while the remaining 68 enterprises are not in default.

Then, the corresponding data of the indicators are analysed. For return on assets, net profit growth rate, asset-liability ratio and other financial indicators, the data used for the calculations can be obtained directly from the financial statements of enterprises. This article obtains the values of these indicators from the Guotai'an database. However, other indicators that are not easy to quantify, such as the degree of information sharing and the degree of dependence of upstream and downstream enterprises, are vague and do not have specific associated data. Most of the current rating companies and commercial banks in credit rating for enterprises use expert evaluation to quantify the qualitative indexes, namely, for each index of evaluation content and evaluation standard, according to the rating object that has reached the level of a given corresponding score, experts assign points to obtain a quantitative score. This article uses this method to quantify qualitative indicators. Each index is divided into five grades of 1, 2, 3, 4, and 5 according to its merits, and industry researchers from several fund companies are invited to score the indexes of the investigated enterprises. In addition, the qualitative index data obtained by the experts are converted to 0.2, 0.4, 0.6, 0.8, and 1.0 for calculation.

### 5.2. Preliminary Screening of the Indicator System

The number of indexes in the index system established in this article is relatively large, and there may be multiple linear problems. Moreover, there is a large amount of sample data corresponding to the indicators. If these indicators are not preliminarily screened, the number of calculations required in the model will be increased, and the analysis efficiency will be reduced. Therefore, preliminary screening of the index system is conducted first; then, principal component factors are extracted for subsequent analysis. The specific screening steps are as follows.

First, the selected sample data are preprocessed. Due to the problem of dimensionless indicators, data are generally treated as dimensionless before feature selection so that the features representing different attributes can be compared. If the original index value is used directly in the analysis, the role of an index with a higher value in the comprehensive analysis will be highlighted, and the role of an index with a lower value will be weakened. In addition, data preprocessing can solve the problem of missing or abnormal data.

Then, under the condition that the sample data satisfy the normal distribution assumption, an independent sample *T* test is performed in SPSS. Next, significant differences are assessed according to the degree of homogeneity of variance to form the main indicator set.

Finally, factor analysis is conducted with SPSS for the index system obtained in the previous step to eliminate the multicollinearity among the indicators and reduce the quantity of unnecessary calculations.

The specific screening process is shown in Figure 3.

#### 5.2.1. Data Preprocessing

Analysis of the obtained data indicates that not all indicators have corresponding data, and the data may be lost. On the other hand, financial indicators, such as return on assets and return on equity, have large corresponding data values, whereas the indicators scored by experts are very small. Moreover, the units of data are different, so the same standard cannot be used for analysis. At this point, the data must be preprocessed. First, missing values and outliers are processed to determine whether they should be deleted or supplemented with data, such as the mean values. Next, a standardized and normalized analysis of these data is required to eliminate the influence of the disunity of units and prepare for the subsequent substitution of data into the constructed CNN model.

*(1) Missing Values and Outlier Processing:* The method mainly includes filling and replacing total constants, filling and replacing average attribute values, and normal values of the time before replacement. The second method is selected according to the specific research idea proposed in this article, that is, to use the overall average value of the corresponding data of the index to fill in missing values and replace outliers.

*(2) Normalization of Data:* This article analyses the following two normalization methods.

The first is the min-max standardization method, which involves linear transformation of the original data and maps the data to [0, 1], also known as deviation standardization. The specific transformation method is shown in formula (9).

(9) $$\begin{array}{c} y=\frac{x-\min}{\max-\min}. \end{array}$$

In the above formula, min is the minimum of the sample and max is the maximum of the sample.

The second is the *z* score standardization method, which is a very common standardization method. This standardization method aims to standardize the original data set to have a mean of 0 and variance of 1, close to the standard normal distribution.

The specific calculation method is shown in formula (10).

(10) $$\begin{array}{c} y=\frac{x-u}{\delta }. \end{array}$$

According to the characteristics of the selected financial data, min-max standardization is used to conduct preliminary data processing.

#### 5.2.2. Significance Test of Indicators

Because this article establishes an index system of financial risk early warning for supply chains that contains 29 indicators, to correctly distinguish whether there is a credit risk for a sample enterprise, screening must be performed. To ensure the validity of the model, this article uses the independent sample *T* test method to construct the initial index system for early screening.

Samples of enterprise data are input into SPSS, and significance testing at a confidence level of ninety percent is performed. The results indicate that sales net interest rate, the net interest rate of the cost and 23 indexes, such as whether sample enterprise credit risk, are significant. These factors can be used effectively to distinguish whether a corporation will default. Therefore, these indicators can be included in the principal component analysis.

#### 5.2.3. Selection of Risk Early Warning Evaluation Indicators Based on Principal Component Analysis

*(1) The Premise of Factor Analysis is that Variables are Correlated; Otherwise, the Variables are not Suitable for Factor Analysis*: Therefore, KMO and Bartlett sphericity tests should be performed on the data corresponding to the indicators first to determine whether common factors can be extracted.

The KMO statistic, which reflects the correlation between variables, ranges from 0 to 1: the larger the value is, the stronger the correlation between variables. In contrast, a value below 0.5 indicates that it is not suitable for factor analysis. The Bartlett sphericity test is used to judge whether variables in the correlation coefficient matrix are independent of each other: if they are independent, factor analysis cannot be performed. From a numerical perspective, as long as the value of Sig. is less than 0.05, the hypothesis is not valid, each variable is correlated, and the common factor can be extracted.

Descriptive statistics were calculated for the data in SPSS, and the results are shown in Table 2.

*2. Extract Common Factors*: SPSS software was used for factor analysis. The maximum variance method was used to rotate the component matrix, and the factors were extracted according to whether the eigenvalues were greater than 1. Eigenvalues of factors that are less than 1 do not explain the original variables well and should therefore be discarded.

In this article, principal component analysis was used to extract common factors, and the total variance of the interpretation obtained is shown in Table 3. The gravel map of the principal component analysis is shown in Figure 4.

Table 3 shows that among the 23 variables, 8 components have eigenvalues greater than 1. The data in the second column represent the corresponding characteristic values of these 8 components, which are 4.472, 3.721, 2.860, 2.179, 1.194, 1.079, 1.068, and 1.037, respectively. The data in the third column represent the explanatory rate of each component to the original variable: 19.443%, 16.179%, 12.434%, 9.476%, 5.193%, 4.691%, 4.643%, and 4.510%. The data in the fourth column indicate that these 8 components accumulatively explain 76.569% of the original variables, accounting for most of the information provided by the original 23 indicators. This conclusion is also verified by the rubble diagram of the principal component analysis in Figure 4. Therefore, we can replace the original 23 initial indicator variables with these 8 principal components.

*3. Rotate the Factor:* To see more clearly the interpretation of the 8 principal components on the original index, we need to rotate the factor loading matrix. The rotated factor loading matrix is shown in Table 4.

The first factor in the core enterprise core enterprise, which is composed of core enterprise operating profit margin, return on net assets, and quick ratio, has a high load on the multiple of interest safeguard and indicates that the four variables are highly correlated. These variables reflect the profitability of the core enterprise, so the first common factor is defined as the core enterprise profit ability factor, *F*1. The second factor has a high load on the price stability of pledges, the vulnerability degree of pledges, and the liquidity ability of pledges. These variables reflect the factors of financing assets, so the second factor is called the operation security factor, *F*2. The third factor accounts for the asset-liability ratio, interest guarantee multiple, liquidity ratio, and quick ratio of financing enterprises. These variables represent the level of debt repayment ability of enterprises. Therefore, the third factor can be called the solvency factor of financing enterprises, *F*3. The fourth factor has a high load on the return on assets of financing enterprises, return on net assets of financing enterprises, growth rate of operating income of financing enterprises, and net interest rate of financing enterprises. These variables represent the profitability of financing enterprises; thus, the fourth factor is named the profitability factor of financing enterprises, *F*4. The fifth factor has a high load on the dependence degree, information sharing degree, and cooperation time of upstream and downstream enterprises. These variables reflect the stability and information sharing degree of the supply chain. Therefore, the fifth factor is named the online degree factor of the supply chain, *F*5. The sixth factor has a high load on the default rate of financing enterprises, which reflects the quality of financing enterprises. Therefore, the sixth factor is named the quality factor of financing enterprises, *F*6. The seventh factor places high importance on the net profit growth rate of financing enterprises and reflects the growth capacity of financing enterprises. Therefore, the seventh factor is called the growth capacity factor of financing enterprises, *F*7. The eighth factor has a high load on the inventory turnover rate and receivables turnover rate of financing enterprises, which reflect the operating capacity of financing enterprises. Therefore, the eighth factor is named the operating capacity factor of financing enterprises, *F*8.

*4. Calculate Factor Scores:* Regression was adopted to estimate the factor scoring coefficient. The specific scoring coefficient matrix of each principal component factor is shown in Table 5, which reflects the correlation degree between each independent variable and 8 common factors.

The original 23 indicators are expressed as *X*_1_, *X*_2_,… *X*_23_, and the extracted 8 common factors are expressed as F_1_, F_2_,… F_8_. Thus, the scoring function of the factors, namely, the principal component expression can be written as follows.

*F*_1_ = −0.011 × *X*_1_−0.032×*X*_2_−0.059 × *X*_3_＋0.027 × *X*_4_＋0.011×*X*_5_

＋0.039×*X*_6_−0.010×*X*_7_−0.009×*X*_8_＋0.049×*X*_9_＋0.039×*X*_10_

＋0.001×*X*_11_﹣0.033×*X*_12_＋0.249×*X*_13_＋0.249×*X*_14_﹣0.249×*X*_15_＋0.249×*X*_16_＋0.003×*X*_17_﹣0.012×*X*_18_﹣0.008×*X*_19_＋0.001×*X*_20_﹣0.007×*X*_21_﹣0.007×*X*_22_﹣0.020×*X*_23_

*F*_2_ = −0.050×*X*_1_−0.008×*X*_2_−0.000×*X*_3_＋0.048×*X*_4_−0.025×*X*_5_

＋0.029×*X*_6_＋0.072×*X*_7_＋0.106×X_8_−0.009×*X*_9_＋0.003×*X*_10_

﹣0.059×*X*_11_＋0.093×*X*_12_−0.004×*X*_13_−0.004×*X*_14_＋0.004×*X*_15_−0.004×*X*_16_＋0.421×*X*_17_＋0.295×*X*_18_﹣0.001×*X*_19_＋0.405×*X*_20_﹣0.057×*X*_21_−0.057×*X*_22_﹣0.044×*X*_23_

*F*_3_ = ﹣0.033×*X*_1_−0.068×*X*_2_＋0.087×*X*_3_−0.023×*X*_4_＋0.030×*X*_5_

−0.143×*X*_6_＋0.030×*X*_7_＋0.103×*X*_8_＋0.384×*X*_9_＋0.382×*X*_10_

−0.159×*X*_11_−0.192×*X*_12_＋0.038×*X*_13_＋0.038×*X*_14_﹣0.038×*X*_15_＋0.038×*X*_16_＋0.011×*X*_17_−0.053×*X*_18_＋0.018×*X*_19_＋0.005×*X*_20_−0.018×*X*_21_−0.0018×*X*_22_﹣0.005×*X*_23_

*F*_4_ = 0.334×*X*_1_＋0.335×*X*_2_＋0.281×*X*_3_−0.107×*X*_4_−0.070×*X*_5_

＋0.159×*X*_6_−0.059×*X*_7_＋0.0291×X_8_−0.016×*X*_9_＋0.000×*X*_10_

＋0.127×*X*_11_＋0.059×*X*_12_−0.034×*X*_13_−0.034×*X*_14_＋0.034×*X*_15_−0.034×*X*_16_﹣0.010×*X*_17_＋0.005×*X*_18_−0.103×*X*_19_﹣0.004×*X*_20_＋0.010×*X*_21_＋0.010×*X*_22_﹣0.072×*X*_23_

*F*_5_ = 0.121×*X*_1_＋0.035×X_2_﹣0.064×*X*_3_＋0.034×*X*_4_＋0.020×*X*_5_

−0.029×*X*_6_−0.093×*X*_7_−0.293×*X*_8_−0.033×*X*_9_−0.061×*X*_10_

＋0.085×*X*_11_−0.201×*X*_12_−0.002×*X*_13_−0.002×*X*_14_＋0.002×*X*_15_−0.002×*X*_16_﹣0.167×*X*_17_−0.016×*X*_18_＋0.038×*X*_19_−0.137×*X*_20_＋0.478×*X*_21_＋0.478×*X*_22_＋0.024×*X*_23_

*F*_6_ = −0.048 × *X*_1_−0.092 × *X*_2_＋0.355 × *X*_3_−0.193 × *X*_4_＋0.019 × *X*_5_

＋0.077 × *X*_6_−0.512 × *X*_7_＋0.209 × *X*_8_−0.002 × *X*_9_＋0.021 × *X*_10_

＋0.063 × *X*_11_＋0.251 × *X*_12_−0.016 × *X*_13_−0.016 × *X*_14_＋0.016 × *X*_15_−0.016 × *X*_16_﹣0.083 × *X*_17_＋0.016 × *X*_18_﹣0.221 × *X*_19_﹣0.085 ×*X*_20_＋0.067 × *X*_21_＋0.067 × *X*_22_＋0.438 × *X*_23_

*F*_7_ = −0.122 × *X*_1_−0.128 × *X*_2_−0.129 × *X*_3_＋0.184 × *X*_4_＋0.776 × *X*_5_

＋0.064 × X_6_−0.134 × *X*_7_＋0.267×*X*_8_＋0.054×*X*_9_＋0.062 × *X*_10_

＋0.276 × *X*_11_−0.016 × *X*_12_＋0.010 × *X*_13_＋0.010 × *X*_14_−0.010 × *X*_15_＋0.010 × *X*_16_﹣0.050 × *X*_17_＋0.062 × *X*_18_＋0.180 × *X*_19_﹣0.068 × *X*_20_＋0.024 × *X*_21_＋0.024 × *X*_22_﹣0.121 × *X*_23_

*F*_8_ = −0.026 × *X*_1_＋0.071 × X_2_−0.083 × X_3_﹣0.607 × *X*_4_＋0.023 × *X*_5_

＋0.140 × *X*_6_＋0.035 × *X*_7_＋0.010 × *X*_8_＋0.073 × *X*_9_＋0.076 × *X*_10_

−0.110 × *X*_11_＋0.202 × *X*_12_−0.023 × *X*_13_−0.023 × *X*_14_＋0.023 × *X*_15_−0.023 × *X*_16_−0.023 × *X*_17_−0.020 × *X*_18_＋0.679 × *X*_19_﹣0.026 × *X*_20_＋0.016 × *X*_21_＋0.016 × *X*_22_＋0.011 × *X*_23_

5. Then, the variance contribution rate of each factor is taken as the weight to calculate the factor weighted total score to conduct risk evaluation. The expression is as follows.

*F*=(0.181/0.765) × F_1_＋(0.121/0.765) × F_2_＋(0.115/0.765) × F_3_＋(0.108/0.765) × F_4_

＋(0.084/0.765) × F_5_＋(0.061/0.765) × F_6_＋(0.048/0.765) × F_7_

＋(0.047/0.765) × F_8_

According to the calculated *F* value, the risk degree can be divided into 4 categories: an F value greater than 1 indicates very low risk; an *F* value between 0 and 1 indicates low risk; an F value between −1 and 0 indicates high risk; and an *F* value less than −1 indicates very high risk.

6. According to the index attribute and scoring standard of supply chain financial risk, the higher the score of the evaluation index is, the lower the supply chain financial risk level of the credit-granting object is; otherwise, the risk level is high, as shown in Table 6. Therefore, credit decisions can be made according to the variation interval of the *F* value, and corresponding risk management measures can be taken to reasonably avoid risks.

### 5.3. Experimental Process and Result Analysis

First, the corresponding values of the 8 principal components are input into the convolution layer as a variable *X*. After convolution of the first layer, ReLU is activated, max-pooling is performed using a 2 × 2 window, and the output result is updated to *X*. The second step is to take the updated variable as the new input data, conduct the second “convolution-activation-pooling” process and obtain the new variable *X*. The third step is to pass *x* through the fully connected layer and the activation function ReLU and then take the output value as the new input before passing through the second fully connected layer to obtain the final output value and the correct number of predicted results. Then, the optimal parameters are obtained via neural network training.

#### 5.3.1. The Influence of Learning Rate on Prediction Results

A good learning rate is conducive to learning the network parameters and can effectively reduce the loss function. A learning rate that is too small will lead to a small weight update, resulting in slow convergence of the cost function and slow model training. A learning rate that is too high may result in the optimal solution being missed. Therefore, this paper uses the selected data set to perform several tests with different learning rate parameters to obtain the parameter settings that are close to optimal for subsequent training. The initial learning rate is trained on the data set many times on the basis of different iterations. The influence of different initial learning rates on the accuracy of the model prediction results is shown in Table 7.

Comparative analysis of the above experimental results indicates that different learning rate settings lead to different levels of accuracy, which will affect the experimental results. The learning rate should be set within a reasonable range. A too high or too low value will reduce the accuracy of model training. As shown in the table, when the learning rate is 0.01, the accuracy of the training data set is relatively high, so the learning rate can be set to 0.01.

#### 5.3.2. The Impact of the Number of Iterations on the Predicted Results Is Shown in Table 8

When the learning rate is 0.01 and multiple iterations are performed, the accuracy of the prediction is the highest when the number of iterations is 200.

#### 5.3.3. Empirical Results of the Model

On the basis of the above parameter settings, a classification test is conducted on the test data set. The four levels of risk warning correspond to categories 0, 1, 2, and 3, and it can be concluded that the comprehensive accuracy of model prediction is 94.7%. The changes in the accuracy of the prediction and loss function are shown in Figures 5 and 6, respectively.

## 6. Conclusion

The supply chain financial risk early warning index system constructed in this article needs to be improved. After reading the relevant literature, it is found that there is still some deficiency in the research on online supply chain finance, and the research on supply chain financial credit risk in the trade circulation industry is not deep enough, so it may be one sided in the analysis of risk influencing factors that it failed to find all the main influencing factors, resulting in deviation in the analysis. There is another reason, although the data of financial indicators can be obtained directly from the enterprise's financial statements, there are many nonfinancial indicators are not easy to obtain. Therefore, the article only selects some indicators that are easy to collect data and may ignore the relatively important influencing factors, which are not easy to obtain. Therefore, in the future research, we should analyze the supply chain financial risk as deeply as possible, and invest more time in data collection to avoid missing those important factors. The accuracy of the data selected for the risk early warning model needs to be improved. The article selects the data of 80 trade circulation enterprises, which may have some shortcomings. In addition, the selection of nonfinancial index data is not easy, and there are some inaccuracies in expert scoring, which will have a certain impact on the training and prediction of the risk early warning model and may reduce the accuracy of the model prediction. In the following research, we should not only ensure the amount of data but also increase the validity and accuracy of the data.

After reviewing the relevant literature, this article summarizes and analyses the main factors affecting the financial risks of the supply chain of the commercial circulation industry. On this basis, combined with the CNN model, a relatively comprehensive risk warning model is built and then validated by means of several examples. The specific results are as follows.

1. First, the literature on the identification and evaluation methods of supply chain financial risk domestically and abroad is analysed and summarized. The indicator system established in some studies is not sufficient, and logistic regression models are most commonly used; thus, the analysis of indicators may not be comprehensive enough. Therefore, a CNN model is adopted in this study to predict supply chain financial risk. The model can further analyze risk influencing factors and obtain accurate results.
2. By analysing the mode of Internet supply chain finance, it is concluded that the supply chain finance mode based on B2C and third-party payments has an effective role in promoting the development of the commercial circulation industry. The process of the four specific financing modes is sorted, and possible sources of risk are summarized to screen out the financial risk impact indicators of the commercial circulation industry chain and finally establish a relatively comprehensive risk early warning indicator system. Including the business development of enterprise ability, profitability, and debt repayment, the ability of four aspects, for a total of 16 financial indexes, contains cooperation with core enterprise time, the degree of information sharing between supply chain enterprises, and the financing of enterprise performance, for a total of 13 nonfinancial indicators of the commerce financial risk early warning index system of the supply chain. By combining the results of the quantitative and qualitative analyses, combining the theoretical basis with the actual situation in the research process, and combining expert experience with mathematical statistics, the above risk warning indicators can be deeply analysed, and accurate results can be obtained.
3. On the basis of the above index system, combined with the CNN method, the supply chain financial risk warning model of the commercial circulation industry, which includes financial and non-financial indicators, is constructed. CNN models have strong self-adaptation and self-learning abilities. The use of a CNN can make the risk analysis of supply chain finance in the commercial circulation industry more depth, resulting in more accurate risk predictions.
4. The corresponding enterprise data are selected for the constructed model. First, the parameter settings of the CNN model are analysed to optimize the results. Then, the optimal parameter settings are determined, and the analysis results are obtained to prove the validity of the model. The results also show that the risk warning model established in this study has a high prediction accuracy and can provide credible support for the prevention and control of supply chain financial credit risks in practice.

## Figures and Tables

**Figure 1:** Design idea of the index system.

**Figure 2:** Convolutional neural network structure.

**Figure 3:** Flow chart of index screening.

**Figure 4:** Rubble diagram of principal component analysis.

**Figure 5:** Change of accuracy rate.

**Figure 6:** Change of loss function.

**Table 1:** Risk early-warning index system.

First-level index	Second-level index	Third-level index	Index description
Financing enterprise qualification	Profitability	Rate of return on assets	(Total profits + financial expenses)/average total assets
		Return on net assets	Net profit/average balance of shareholders' equity
		Net operating rate	Net profit/operating income
	Management ability	Turnover rate of accounts receivable	Average occupation of operating income/accounts receivable
		Inventory turnover	Operating cost/average inventory occupancy
		Total asset turnover	Operating income/total average assets
	Development ability	Growth rate of operating income	(Operating income for the current period this year - operating income for the same period last year)/operating income for the same period last year
		Net profit growth rate	(Current amount of net profit this year - amount of net profit in the same period last year)/amount of net profit in the same period last year
	Debt-paying ability	Current ratio	Current assets/liabilities
		Quick ratio	(Current assets - inventory)/current liabilities
		Interest protection multiple	(Net profit + income tax expenses + financial expenses)/financial expenses
		Asset-liability ratio	Total liabilities/assets
Operating environment condition	Macroeconomy environment	Macroeconomic operation state	
		National macrocontrol policy	
		Legal and policy environment	
	Industry development prospect	Industrial policy	
		Industry development stage	
		Industry competition intensity	
Core enterprise qualification	Profitability	Return on net assets	Net profit/average balance of shareholders' equity
		Operating profit margin	Operating profit/operating income
	Debt-paying ability	Quick ratio	(Current assets - inventory)/current liabilities
		Interest protection multiple	(Net profit + income tax expenses + financial expenses)/financial expenses
	Material characteristics	Price stability	Price fluctuation range of pledged goods in the last quarter
		Cash ability	The ability to sell pledged goods for cash
		The material is easy to be damaged. Degree	The natural property of the material and whether it is conducive to preservation
Supply chain Operation condition	Close cooperation degree	Cooperation time	Year of cooperation between core enterprises and financing enterprises
		Degree of information sharing	Information sharing degree of B2C supply chain
	Upstream and downstream enterprises Degree of dependence		The degree of connection between the financing enterprise and the core enterprise
	Previous performance situation	Financing enterprise Breach of contract record	Whether to breach the contract or not

**Table 2:** KMO and Bartlett sphericity test.

KMO and Bartlett test		
KMO sampling appropriateness quantity		0.820
Bartlett sphericity test	Approximate chi-square	937.920
	Degree of freedom	153
	Significance	0.000

It can be seen from the test results that the value of KMO is 0.82, the Sig of Bartlett's sphericity test. The value is 0, which meets the condition of factor analysis.

**Table 3:** Percent of total variance explained.

Total variance interpretation									
Initial eigenvalue				Extract the sum of squares of load			Sum of squares of rotating load		
Composition	Total	Percentage of variance	Cumulative%	Total	Percentage of variance	Cumulative%	Total	Percentage of variance	Cumulative%
1	4.472	19.443	19.443	4.472	19.443	19.443	4.171	18.133	18.133
2	3.721	16.179	35.622	3.721	16.179	35.622	2.776	12.072	30.205
3	2.860	12.434	48.057	2.860	12.434	48.057	2.642	11.488	41.693
4	2.179	9.476	57.532	2.179	9.476	57.532	2.473	10.750	52.444
5	1.194	5.193	62.725	1.194	5.193	62.725	1.941	8.440	60.883
6	1.079	4.691	67.416	1.079	4.691	67.416	1.404	6.104	66.987
7	1.068	4.643	72.059	1.068	4.643	72.059	1.112	4.837	71.824
8	1.037	4.510	76.569	1.037	4.510	76.569	1.091	4.745	76.569
9	0.952	4.139	80.708						
10	0.911	3.962	84.669						
11	0.819	3.561	88.230						
12	0.762	3.312	91.542						
13	0.625	2.718	94.260						
14	0.504	2.191	96.451						
15	0.417	1.813	98.264						
16	0.309	1.344	99.608						
17	0.052	0.227	99.835						
18	0.032	0.141	99.976						
19	0.005	0.024	100.000						
20	2.780*E* − 15	1.209*E* − 14	100.000						
21	1.539*E* − 16	6.690*E* − 16	100.000						
22	−1.522*E* − 16	−6.618*E* − 16	100.000						
23	−2.478*E* − 15	−1.077*E* − 14	100.000						

Extraction method: Principal component analysis.

**Table 4:** Rotation of the component matrix.

Composition								
	1	2	3	4	5	6	7	8
Operating profit margin of core enterprises	0.993	0.009	-0.065	0.041	0.001	0.029	−0.031	0.018
Return on net assets of core enterprises	0.993	0.009	−0.065	0.041	0.001	0.029	−0.031	0.018
Quick ratio of core enterprises	0.993	−0.009	0.065	−0.041	−0.001	−0.029	0.031	−0.018
Interest guarantee multiple of core enterprise	0.993	0.009	−0.065	0.041	0.001	0.029	−0.031	0.018
Price stability of pledged goods	0.023	0.958	0.065	−0.020	0.119	0.015	−0.031	0.005
Vulnerability of pledged goods	0.023	0.944	0.061	−0.004	0.159	0.007	−0.050	0.004
Liquidity of pledged property	−0.001	0.795	−0.069	−0.007	0.268	0.107	0.090	0.012
Liquidity ratio of financing enterprises	−0.038	0.045	0.955	0.064	0.075	0.015	0.025	0.049
Quick ratio of financing enterprises	−0.071	0.055	0.952	0.080	0.038	0.038	0.037	0.050
Asset-liability ratio of financing enterprises	0.090	0.098	0.540	−0.094	−0.308	0.330	−0.011	0.236
Total asset turnover of financing enterprises	0.352	0.061	0.389	0.341	−0.026	0.030	0.096	0.174
Interest guarantee multiple of financing enterprise	0.106	−0.087	0.383	0.315	0.067	−0.021	0.336	−0.109
Rate of return on assets of financing enterprises	0.122	−0.046	0.029	0.842	0.223	−0.252	−0.070	−0.026
Rate of return on net assets of financing enterprises	0.071	−0.037	−0.082	0.834	0.091	−0.310	−0.070	0.074
Growth rate of operating income of financing enterprises	0.018	0.085	0.241	0.611	−0.335	0.118	0.332	−0.015
Net operating interest rate of financing enterprise	−0.130	0.046	0.325	0.456	−0.010	0.333	−0.114	−0.101
Degree of dependence of upstream and downstream enterprises	0.003	0.376	0.123	0.077	0.871	0.118	0.028	0.055
Degree of information sharing	0.003	0.376	0.123	0.077	0.871	0.118	0.028	0.055
Cooperation time	−0.128	−0.067	0.048	0.100	0.662	−0.156	−0.123	0.015
Default rate of financing enterprises	−0.037	0.043	0.002	−0.449	0.031	0.648	−0.177	0.029
Growth rate of net profit of financing enterprises	−0.104	0.013	0.012	−0.030	0.024	0.011	0.845	0.008
Inventory growth rate of financing enterprises	−0.014	0.057	−0.031	−0.102	0.098	−0.231	0.182	0.728
Turnover rate of accounts receivable of financing enterprises	−0.083	0.043	−0.037	−0.102	0.016	−0.228	0.213	0.658

**Table 5:** Factor scoring coefficient matrix.

Composition								
	1	2	3	4	5	6	7	8
Rate of return on assets of financing enterprises	−0.011	−0.050	−0.033	0.334	0.121	−0.048	−0.122	−0.026
Rate of return on net assets of financing enterprises	−0.032	−0.008	−0.068	0.335	0.035	−0.092	−0.128	0.071
Net operating interest rate of financing enterprise	−0.059	0.000	0.087	0.281	−0.064	0.355	−0.129	−0.083
Turnover rate of accounts receivable of financing enterprises	0.027	0.048	−0.023	−0.107	0.034	−0.193	0.184	−0.607
Inventory turnover of financing enterprises	0.011	−0.025	0.030	−0.070	0.020	0.019	0.776	0.023
Inventory turnover of financing enterprises	0.039	0.029	−0.143	0.159	−0.029	0.077	0.064	0.140
Growth rate of net profit of financing enterprises	−0.010	0.072	0.030	−0.059	−0.093	−0.512	−0.134	0.035
Growth rate of operating income of financing enterprises	−0.009	0.106	0.103	0.291	−0.293	0.209	0.267	0.010
Liquidity ratio of financing enterprises	0.049	−0.009	0.384	−0.016	−0.033	−0.002	0.054	0.073
Quick ratio of financing enterprises	0.039	0.003	0.382	0.000	−0.061	0.021	0.062	0.076
Interest guarantee multiple of financing enterprise	0.001	−0.059	−0.159	0.127	0.085	0.063	0.276	−0.110
Asset-liability ratio of financing enterprises	−0.033	0.093	−0.192	0.059	−0.201	0.251	−0.016	0.202
Return on net assets of core enterprises	0.249	−0.004	0.038	−0.034	−0.002	−0.016	0.010	−0.023
Operating profit margin of core enterprises	0.249	−0.004	0.038	−0.034	−0.002	−0.016	0.010	−0.023
Quick ratio of core enterprises	−0.249	0.004	−0.038	0.034	0.002	0.016	−0.010	0.023
Interest guarantee multiple of core enterprise	0.249	−0.004	0.038	−0.034	−0.002	−0.016	0.010	−0.023
Price stability of pledged goods	0.003	0.421	0.011	−0.010	−0.167	−0.083	−0.050	−0.023
Liquidity of pledged property	−0.012	0.295	−0.053	0.005	−0.016	0.016	0.062	−0.020
Degree of vulnerability of materials	−0.008	−0.001	0.018	−0.103	0.038	−0.221	0.180	0.679
Cooperation time	0.001	0.405	0.005	−0.004	−0.137	−0.085	−0.068	−0.026
Degree of information sharing	−0.007	−0.057	−0.018	0.010	0.478	0.067	0.024	0.016
Degree of dependence of upstream and downstream enterprises	−0.007	−0.057	−0.018	0.010	0.478	0.067	0.024	0.016
Default rate of financing enterprises	−0.020	−0.044	−0.005	−0.072	0.024	0.438	−0.121	0.011

**Table 6:** Corresponding table of early warning levels of supply chain financial risk indicators.

Evaluation index value	*F* > 1	0<*F* < 1	−1<*F* < 0	*F* < −1
Risk level	Low	Lower	Higher	High
Early warning level	Safety	Be careful	Alert	Danger

**Table 7:** Influence of different learning rates on prediction accuracy.

Learning rate	Prediction accuracy (%)
0.5	55.6
0.3	57.6
0.1	86.1
0.01	95.6
0.001	93.3
0.0001	86.2

**Table 8:** Influence of different numbers of iterations on the prediction accuracy.

Number of iterations	Prediction accuracy (%)
10	50.3
50	88.7
100	90
150	93.3
200	96
250	94
300	91.3

## Data Availability

The data come from a survey of China's trade circulation industry. The data used to support the findings of this study are available from the corresponding author upon request.
